# Antiplasmodial Activity of 80% Methanolic Extract and Solvent Fractions of Stem Bark of *Acacia tortilis* in Swiss Albino Mice

**DOI:** 10.1155/2022/7493294

**Published:** 2022-11-04

**Authors:** Muluken Adela Alemu, Yared Andargie Ferede, Getu Tesfaw Addis, Sintayehu Asnakew Alemayehu, Tewodros Ayalew Tessema, Rahel Belete Abebe, Getaye Tessema Desta, Yohannes Shumet Yimer

**Affiliations:** ^1^Department of Pharmacy, Debre Tabor University, Debre Tabor, Amhara, Ethiopia; ^2^Department of Nursing, Debre Tabor University, Debre Tabor, Amhara, Ethiopia; ^3^School of Pharmacy, University of Gondar, Gondar, Amhara, Ethiopia

## Abstract

**Background:**

Malarial infection has significant negative impact on the health of the world population. It is treated by modern and traditional medicines. Among traditional medicinal plants, *Acacia tortilis* is used by different communities as antimalarial agent. Therefore, the objective of this study is to validate antimalarial activity of the stem bark of *Acacia tortilis* in mice.

**Methods:**

To evaluate antimalarial activity of the plant, 4-day suppressive, curative, and prophylactic antimalarial test models were used. Parasitemia, packed cell volume (PCV), survival time, rectal temperature, and body weight were used to evaluate the effect of the plant extracts. Data were analyzed using SPSS version 26 followed by Tukey's post hoc multiple comparison test.

**Results:**

The crude extract and dichloromethane fraction significantly suppressed the level of parasitemia (*p* < 0.001) and increased mean survival time (*p* < 0.01) at all tested doses. Similarly, significant effects were observed in mean survival time, % change of PCV, weight, and temperature in both curative and prophylactic antimalarial test models.

**Conclusions:**

The methanolic extract and solvent fractions of the stem bark of *Acacia tortilis* has shown antimalarial activity, and the finding supports the traditional use and the *in vitro* studies. Thus, this study can be used as an initiation for researchers to find the most active phytochemical entity and to conduct additional safety and efficacy tests.

## 1. Introduction

Malarial infection has a significant negative impact on the health of the world population [1]. Higher deaths were enumerated in under-five children in sub-Saharan Africa where infectious diseases are still the primary public health concern [2, 3]. Children and pregnant women are selectively affected by malaria. In 2019, malaria was responsible for the death of 409,000 people. Of these 94% deaths occurred in Africa and the death of young children accounts for a total of 274,000 [4]. Children who recovered from cerebral malaria (2%) develop several disabilities and impairments [5]. In 2020, it is estimated that 215.2 million cases and 386,400 deaths in malaria-endemic countries in Africa [6].

According to 2019 World Health Organization estimation, the incidence of malaria was 229 million of which 409, 000 deaths were registered in the world while the most (94%) was in the African region [7]. Apart from death, the disease results serious complications like cerebral malaria, severe anemia, hypoglycemia, and acute renal failure [8, 9].

In 2020, a year after the COVID-19 pandemic, the number cases of malaria rose to 241 million, an increment of 12 million cases as of 2019. In the African region, between 2019 and 2020, the cases of malaria had grown from 213 to 228 million and deaths from 534 000 to 602, 000 between 2019 and 2020. The region has valued 95% and 96% global cases and deaths, respectively, among which the deaths of under-five children accounted 80% [10].

A single antimalarial drug is not effective for both stages (liver and intra-erythrocytic) of malaria parasite. Due to this many drugs may be used to have complete elimination of a parasite from the already established infection [11].

*Acacia* tortilis (*Fabaceae* family) is a slow growing tree having an umbrella-shaped canopy [12]. Traditionally, the plant has inspiring medicinal uses for mouth infections and dental problems [13], dry cough, and diphtheria [14]. It has been proved that it contains antidiabetic [15], antifungal [16], antidiarrheal [17], antihyperlipidemic [18], anti-inflammatory [19], antimalarial, and antileshmanial [20] activities. Similarly, the whole plant [21] and the stem bark [22] of *Acacia tortilis* showed very active and active *in vitro* antiplasmodial activities, respectively. Resistance to artemisinin antimalarial drugs was reported in murine malaria models [23] and in patients on the Cambodia-Thailand border [24]. So, there is a need to validate the *in vitro* antimalarial activity in mice model and innovate new drugs to fill the resistance problem. Therefore, this study was aimed to investigate antimalarial activity of the plant in the rodent model and ensure which solvent fraction(s) is/are more effective so that a clue about the nature of the effective phytochemical constituents can be obtained.

## 2. Materials and Methods

### 2.1. Plant Material

The stem bark of the plant was collected from Makisegnit Woreda, Central Gondar, Amhara, Ethiopia in November 2021. Identification and authentication was made by a botanist and a voucher specimen number was given (MA03).

### 2.2. Experimental Animals and Parasite

Swiss albino mice weighing 20 to 30 g, aged 6 to 8 weeks (males for antimalarial test and females for acute oral toxicity test) were selected and used. The mice were given free access to pelleted food and water. They were kept in a standard plastic cage at room temperature and light having a cycle of 12 h light and 12 h dark. The mice were acclimatized to the laboratory class 7 days prior to the start of the experiment. *Plasmodium berghei* strain which is chloroquine sensitive was used for the antimalarial test. The continuity of the parasite was ensured by transferring blood from infected to noninfected mice weekly.

Animals were handled based on the internationally accepted guidelines for care and use of animals. Ethical issues and the study protocol were approved by the ethical committee.

### 2.3. Extraction and Fractionation

The stem bark was first cleaned and then dried under shade. The dried bark was grounded into small pieces using mortar and pestle. About 1.5 kg coarse powder of the bark was weighed by Wensar analytical balance (Swastic Systems and Services, India) and then extracted with the cold maceration technique. Then, No 1 Whatman filter paper was used to filter the extract. The mark was re-extracted two times by adding similar volume of the fresh solvent. The filtrates added together and were allowed to be concentrated at a temperature less than 40°C. The concentrated extract was then frozen and dried using a lyophilizer. The dried extract was then fractionated using hexane, dichloromethane, and water. Initially, the crude extract was mixed with water and then shaken using a separatory funnel. Hexane was added three times separately to get a hexane fraction. Then, dichloromethane was added to the residue three times and then dichloromethane filtrate was obtained. The extracts were concentrated using a rotary evaporator. The aqueous residue was dried using a lyophilizer. Finally, the crude extract and the fractions were stored at −20°C until being used for the experiment.

### 2.4. Phytochemical Screening of the Stem Bark of *Acacia tortilis*

Both the crude extract fractions were screened for the presence or absence of secondary metabolites such as tannins, flavonoids, anthraquinones, glycosides, phenols, steroids, terpenoids, alkaloids, and saponins using standard screening tests [25].

### 2.5. Acute Oral Toxicity Test

Acute toxicity test for the crude extract was performed based on the guideline 420 developed by the Organization for Economic Co-operation and Development (OECD) [26]. Female mice with the age 6 to 8 weeks were used for the test. They were fasted 4 h before and 2 h after administration of the crude extract. Initially, sighting study was performed to determine the starting dose by administering 2000 mg/kg of the extract to a single mouse. Since no sign of toxicity and death was observed in 24 h, the same dose was given to 4 mice through oral gavage. The presence of toxicity, death, and food intake was strictly followed for 4 h and then for 14 days.

### 2.6. Grouping and Dosing

Animals were randomly assigned into 5 groups (6 animals per group) for each model. Group I (negative control) received 10 ml/kg of the dissolving vehicle (2% tween 80 for hexane and dichloromethane fractions and 10 ml/kg distilled water for the crude extract and distilled water fraction). Group II received the positive control, and the groups from III to V received 100 mg/kg, 200 mg/kg, and 400 mg/kg of the crude extract and fractions.

### 2.7. Inoculation

First, the level of parasitemia for the donor mice was determined (20%–30%). After ether anesthesia, mice were sacrificed through cervical dislocation and then blood was taken by cardiac puncture and collected in a heparinized tube. The blood was diluted with normal saline (0.9%) to the level of 5 × 10^7^ of infected red blood cell (RBC) in 1 ml. Each mouse was given 0.2 ml of blood (containing 1 × 10^7^ infected RBCs) intraperitoneally.

## 3. Determination of Antimalarial Activity

### 3.1. Four-Day Suppressive Test

Peter's suppressive test method was used to assess the chemo-suppressive effect of the plant extracts against chloroquine sensitive *P. berghei* [27]. Prior to infection, the weight of mice, packed cell volume (PCV), and temperature were measured. Then, thirty mice for the crude extract and each of solvent fractions were parasitized on the first day (day 0). Two hour later, mice were randomly grouped into 5 groups and given doses as indicated in the grouping and dosing section. Treatment doses were continued being given at 24, 48, and 72 h (until the third day). On the fourth day of infection (96 h later), blood was taken from the tail of each mouse and then the parasitemia level and percentage chemosuppression was determined by preparing thin smears on the microscope slides. At the end of the experiment, the weight of mice, packed cell volume (PCV), and temperature were measured. Then, the mean survival time was evaluated by following the mice for 30 days (day 0 to day 29).

### 3.2. Curative Test

The curative test was conducted for the crude extract and dichloromethane fraction, which have shown relatively higher parasitemia suppression in a four-day suppression test. The curative potential of the plant in an established infection was conducted using the method indicated by Raley and Peters [28]. For each test extract, thirty mice were infected on the first day (day 0). After day 3 (72 h), mice were grouped into five groups (six per group) and treated with respective doses of the crude extract and dichloromethane fraction as indicated in the grouping and dosing section. Treatment doses were continued to be given at 96, 120, and 144 h. The level of parasitemia was recorded daily from day 3 to day 6. The weight of mice, packed cell volume (PCV), temperature, and survival time were also recorded.

### 3.3. Prophylactic Test

The prophylactic effect of the crude extract and dichloromethane fraction was done as indicated by Peters et al. [27]. For both of the extracts, mice (thirty for each) were randomly assigned to five groups and treated as pointed in the grouping and dosing section. Treatment was consecutively given daily for four days and all mice were intraperitoneally infected with the parasite (1 × 10^7^*P. berghei*) on the 5th day. Blood smears were prepared 72 h after infection and the parasitemia level was determined. In addition, the weight of mice, temperature, packed cell volume (PCV), and survival time were also recorded.

### 3.4. Determination of Parasitemia and Survival Time

Blood smears from each mouse were applied on different microscope slides and then were fixed with methanol. Then, the slides were stained with 10% Geimsa stain for 15 min and were washed with water and then dried at room temperature. Finally, parasite-infected RBCs were counted using microscope having a magnification power of 100x. The level of parasitemia was calculated by the experiment blinded laboratory technician. % Parasitemia was computed by enumerating the infected RBC and total RBC from the blood films while parasitemia suppression was calculated by comparing parasitemia in the negative control with parasitemia in the treated group with the following formulas [29]:

(1) $$\begin{array}{c} \%\;Parasitemia=\frac{Number\;of\;parasitize\;d\;RBC}{Total\;number\;of\;counte\;d\;RBC}\times 100,\%\;Chemosuppresion=\frac{Mean\;parasitemia\;in\;treate\;d\;group}{Mean\;parasitemia\;in\;negative\;control\;group\;}\times 100. \end{array}$$

At last, mice were followed for 30 days (from day 0 to day 29) and their mean survival time (MST) was determined as indicated in the following formula [29]:

(2) $$\begin{array}{c} MST=\frac{Total\;number\;of\;da\;ys\;mice\;survive\;d}{Total\;number\;of\;mice}\text{.} \end{array}$$

### 3.5. Determination of Packed Cell Volume, Rectal Temperature, and Body Weight

Blood was taken from the tail of each mouse and was collected in heparinized microhaematocrit capillary tubes to 75% of their height and then was sealed. The tubes were then placed on a centrifuge and were rotated at 12,000 rpm for 5 min. Packed cell volume (PCV) was computed through the following formula [30]:

(3) $$\begin{array}{c} PCV=\frac{Volume\;of\;erythrocytes\;in\;a\;given\;volume\;of\;bloo\;d}{Total\;bloo\;d\;volume}\times 100. \end{array}$$

The weight of each mouse was measured using the weighing balance, and rectal temperature was tested using the rectal thermometer. The changes before and after treatment were then calculated.

### 3.6. Data Analysis

The data were analyzed using SPSS version 25. The results were expressed as mean ± SEM (standard error of the mean). One-way ANOVA and Tukey's post hoc test for comparisons were used to compare differences in the groups. Results were considered significant at 95% confidence level at *P* value < 0.05.

## 4. Results

### 4.1. Yields of the Crude Extract and Solvent Fractions

After extracting 1.5 kg of the stem bark with 80% methanol, 121 g of the crude extract was obtained. Upon fractionation of 90 g of the crude extract, 65 g, 15.5 g, and 9.5 g of water, dichloromethane, and hexane fractions were obtained, respectively.

### 4.2. Phytochemical Screening

The extract of the stem bark was screened for the availability of different phytochemicals. Based on this, many phytochemicals were present in the crude extract and were proved to be attracted to dichloromethane as indicated in Table 1.

### 4.3. Acute Oral Toxicity Test

The crude extract of the stem bark of *Acacia tortilis* at 2000 mg/kg dose did not show any sign of toxicity or death in the 14-day follow-up period. No visible adverse effects like changes in feeding, body weight, hair erection, urination, lacrimation, salivation, and movement were observed, indicating the extract is safe.

## 5. Determination of Antimalarial Activity

### 5.1. Effects of the Crude Extract and Solvent Fractions of the Stem Bark of *Acacia tortilis* in the 4-Day Suppressive Test

The crude extract and dichloromethane fraction produced significant differences on the parasitemia level and mean survival time at all tested doses as compared to the negative control. In addition, the aqueous fraction showed a meaningful difference on the parasitemia level (at 400 mg/kg dose) and mean survival time (at 200 and 400 mg/kg doses), while the hexane fraction revealed a significant difference at 400 mg/kg dose on mean survival time (Table 2). The activity of both the crude extract and solvent fractions increased as the dose increases.

As indicated in Table 3, the crude extract produced a meaningful effect on the % change of packed cell volume (PCV) (400 mg/kg), temperature change (200 and 400 mg/kg), and weight change at all tested doses. Aqueous fraction produced significant differences on temperature and weight change at 400 mg/kg dose. In addition, dichloromethane fraction (at all tested doses) produced significant effects on % changes of PCV, temperature, and weight; but hexane fraction showed significant activities only on temperature change at 200 and 400 mg/kg doses. The activities for all the extracts increase as the dose increases indicating the effects are dose dependent.

### 5.2. Effects of the Crude Extract and Dichloromethane Fraction of the Stem Bark of *Acacia tortilis* in the Curative Test Model

The crude extract and dichloromethane fraction has shown a relatively greater antimalarial activity in the 4-day suppressive test. Therefore, these extracts are selected for further evaluation in curative and prophylactic antimalarial test models.

Both the crude extract and the dichloromethane fraction revealed significant effects on % parasitemia from day 5 to day 7 (Table 4). Similarly, both the crude extract and the fraction showed a meaningful difference on mean survival time as compared to the negative control at all tested doses (*p* < 0.001). The activities of each extract increased as the dose increases.

As shown in Table 5, the crude extract produced significant difference on the % change of PCV and rectal temperature (at 200 and 400 mg/kg) as well as body weight at 400 mg/kg dose. In addition, dichloromethane fraction produced a meaningful difference on % change of the weight and rectal temperature at all tried doses in a dose-dependent manner (*p* < 0.001), while a significant effect on the % change of body weight was observed at 400 mg/kg dose (*p* < 0.05).

### 5.3. Effects of the Crude Extract and Dichloromethane Fraction of the Stem Bark of *Acacia tortilis* in the Prophylactic Test Model

In comparison with the negative control, both the crude extract and dichloromethane fraction showed significant effects on both the % parasitemia (*p* < 0.001) and mean survival time (*p* < 0.01) at all tested doses (100, 200, and 400 mg/kg). Both of the extracts showed comparable effects on % suppression and mean survival time (Table 6).

As compared to the negative control, significant differences on the % change of PCV, rectal temperature, and body weight were seen at 400 mg/kg dose of both the crude extract and dichloromethane fraction. Dichloromethane fraction produced relatively higher activities than the crude extract on the tested parameters (Table 7).

## 6. Discussion

The current treatment of malaria gets serious challenges due to the emergence of resistance to the available drugs and unavailability of vaccines [31, 32]. Malaria caused by *P. falciparum* is a serious disease, if untreated, it may progress to being life threatening and then result in death [33]. Therefore, there is a need to find new medicines from different sources.

The extracts of *Acacia tortilis* were evaluated for their acute oral toxicity and antimalarial activities in three rodent test models. Using rodents for testing antimalarial activity of the compounds is important since it can show the activity of prodrugs that need activation in living systems unlike *in vitro* studies [34]. Therefore, the rodent malaria model was used to test the antimalarial activity of the plant extract. The crude extract of the plant did not show any toxicity signs at a dose of 2000 mg/kg. Accordingly, this extract can be considered good for further studies since the LD_50_ is above 20 times the minimum tried effective dose (100 mg/kg) [35].

The antimalarial activities of the crude extract and solvent fractions of *Acacia tortilis* were evaluated using standardized models. Accordingly, the 4-day suppressive test was conducted for evaluating schizontocidal activity at the start of the infection while the curative test was employed to assess curative potential of the extracts on an already established infection, and the prophylactic test was done to assess the infection preventive activity of the plant [36]. According to the category of biological substances, the study result showed the extract is endowed with antimalarial activity and the result was in line with the previous very active and active *in vitro* antiplasmodial activities of the whole plant and the bark, respectively [21, 22, 37].

An extract with greater than 30% suppressive effect (as compared to the negative control) on the level of parasitemia is considered as effective [38]. As shown in Table 2, in the 4-day suppressive test, both the crude extract and dichloromethane fraction showed parasitemia suppression at all tested doses (*p* < 0.001) confirming the probable schizontocidal effect. All the tested doses of the extract revealed an increase in the mean survival time explaining the associated decrease in the parasitemia level. This result is in line with the study conducted on *Croton macrostachys* [39]. In addition, the better activity of the dichloromethane fraction on the % change of PCV, temperature, and weight was in line with the very active *in vitro* antiplasmodial activity of the dichloromethane extract of the plant. The difference in the activity may be due to the variation in the presence of secondary metabolites in the fractionating solvents. In addition, variation in the concentration of secondary metabolites in the fractionating solvents may account for the activity difference.

In the curative test, significant suppression on the parasitemia level was observed at all tested doses of both the crude extract and dichloromethane fraction, indicating the effect of the extract on the established infection. In this model, antimalarial activity was tested for the crude extract and dichloromethane fraction, since they showed better activity in the 4-day suppressive test model in a dose-dependent manner.

After confirming the positive curative effect, the evaluation was continued to validate the prophylactic effect of the plant. In the study, the crude extract and dichloromethane fraction had shown a chemoprophylactic effect in a dose-dependent manner. Several secondary metabolites like alkaloids and flavonoids were screened in both the crude extract and dichloromethane fraction. Secondary metabolites are implicated in antiplasmodial activities through different mechanisms. Alkaloids are known to possess antimalarial activity [40]. Saponins, flavonoids, and terpenoids may be responsible for the observed antimalarial activity [41]. In addition, secondary metabolites are involved in several functions including endoperoxidation by terpenoids [42], DNA intercalation by anthraquinones [43], disruption of detoxification of heme by alkaloids [44], inhibition of protein synthesis by alkaloids and disruption of nucleic acids by flavonoids [45], inhibition of superoxide dismutase and inhibition of DNA synthesis by coumarins [46], and free radical scavenging by tannins [47]. Furthermore, glycosides are known to have a direct antiplasmodial effect [48]. The observed antimalarial effect may be due to the in concert effect of these secondary metabolites.

## 7. Conclusions

The methanolic extract and solvent fractions of the stem bark of *Acacia tortilis* has shown antimalarial activity, and the finding supports the traditional use and the *in vitro* studies. Thus, this study can be used as an initiation for researchers to find the most active phytochemical entity and to conduct additional safety and efficacy tests.

## Figures and Tables

**Table 1:** Phytochemical screening of the crude extract and solvent fractions of the stem bark of *Acacia tortilis*.

Phytochemical constituents	Crude extract	Fractions		
		Water fraction	Dichloromethane fraction	Hexane fraction
Alkaloids	+	+	+	—
Anthraquinones	+	+	+	—
Cardiac glycosides	—	—	—	—
Flavonoids	+	—	+	+
Glycosides	+	+	—	—
Phenols	+	+	+	—
Saponins	+	+	+	—
Steroids	+	—	—	+
Tannins	+	+	+	—
Terpenoids	+	—	+	+

Keys: + present, — absent.

**Table 2:** Effects of crude extract and solvent fractions of *Acacia tortilis* on the parasitemia level and mean survival time in the 4-day suppressive test.

Treatment and doses	% Parasitemia	% Suppression	Mean survival time (days)
10 ml/kg DW	31.83 ± 1.17	0.00	6.00 ± 0.58
CHQ 25 mg/kg	0.00 ± 0.00^a3^	100.00	30.00 ± 0.00^a3^
100 mg/kg CE	19.67 ± 1.52^a3,b3^	38.20	9.17 ± 0.60^a2,b3,e3^
200 mg/kg CE	18.33 ± 1.23^a3,b3^	42.41	11.17 ± 0.60^a3,b3,e3^
400 mg/kg CE	15.50 ± 0.67^a3,b3^	51.30	15.00 ± 0.58^a3,b3^
100 mg/kg AF	29.67 ± 1.05^b3,e2^	6.79	7.33 ± 0.42^b3,e3^
200 mg/kg AF	28.50 ± 0.76^b3,e1^	10.46	8.33 ± 0.80^a1,b3,e2^
400 mg/kg AF	24.50 ± 1.06^a1,b3^	23.03	11.33 ± 0.49^a2,b3^
10 ml/kg 2% *T* 80^*∗*^	31.33 ± 1.05	0.00	6.67 ± 0.67
CHQ 25 mg/kg^*∗*^	0.00 ± 0.00^a3^	100.00	30.00 ± 0.00^a3^
100 mg/kg DF	22.67 ± 1.17^a3,b3,d1,e3^	27.64	9.00 ± 0.82^a2,b3,d3,e3^
200 mg/kg DF	17.50 ± 1.26^a3,b3^	44.14	15.50 ± 1.12^a3,b3,c3^
400 mg/kg DF	13.67 ± 0.99^a3,b3^	56.37	17.33 ± 1.11^a3,b3,c3^
100 mg/kg HF	30.17 ± 1.47^b3^	3.70	7.67 ± 0.49^b3,e1^
200 mg/kg HF	28.33 ± 0.88^b3^	9.58	8.00 ± 0.58^b3^
400 mg/kg HF	27.50 ± 0.99^b3^	12.22	10.17 ± 0.87^a1,b3^

Data are expressed as mean ± SEM; *n* = 6, a = compared to the negative control, b = compared to the positive control, c = compared to 100 mg/kg, d = compared to 200 mg/kg, e = compared to 400 mg/kg, ^1^*p* < 0.05, ^2^*p* < 0.01, ^3^*p* < 0.001, ^*∗*^ = negative and positive controls for dichloromethane and hexane fractions, SEM = standard error of the mean, *D*0 = day 0, *D*4 = day 4, DW = distilled water, CE = crude extract, AF = aqueous fraction, DF = dichloromethane fraction, HF = hexane fraction, *T*80 = tween-80, and CHQ = chloroquine.

**Table 3:** Packed cell volume (PCV), weight, and temperature for the crude extract and solvent fractions of the stem bark of *Acacia tortilis* in the 4-day suppressive test.

Treatment	PCV			Temperature (°C)			Body weight (g)		
	PCV at D0	PCV at D4	% PCV change	T° at D0	T° at D4	% T° change	Weight at D0	Weight at D4	% Weight change
10 ml/kg DW	54.83 ± 1.40	44.67 ± 1.54	−18.41 ± 2.82	36.73 ± 0.05	34.23 ± 0.24	−6.80 ± 0.70	24.67 ± 1.28	22.00 ± 1.13	−10.78 ± 0.59
CHQ 25 mg/kg	56.50 ± 0.76	55.67 ± 0.67^a3^	−1.46 ± 0.29^a3^	36.42 ± 0.10	36.43 ± 0.08^a3^	0.05 ± 0.19^a3^	23.67 ± 1.41	23.50 ± 1.26	−0.56 ±0.56^a3^
100 mg/kg CE	54.33 ± 0.67	46.67 ± 1.61^b2^	−14.20 ± 2.09^b2^	36.40 ± 0.14	34.45 ± 0.12^b3^	−5.35 ± 0.59^b3^	26.17 ± 1.11	25.17 ± 0.91	−3.65 ± 1.31^a3^
200 mg/kg CE	52.83 ± 0.48	47.67 ± 1.61^b2^	−9.72 ± 3.23	36.47 ± 0.11	34.97 ± 0.35^b3^	−4.12 ± 0.68^a1,b3^	24.50 ± 1.52	23.67 ± 1.31	−3.15 ± 1.15^a3^
400 mg/kg CE	53.67 ± 0.80	50.83 ± 0.95^a1^	−5.17 ± 2.26^a2^	36.13 ± 0.09	34.93 ± 0.15^b3^	−3.32 ± 0.33^a3,b2^	25.00 ± 0.97	24.33 ± 0.84	−2.58 ± 0.82^a3^
100 mg/kg AF	55.17 ± 0.83	46.83 ± 1.17^b3^	−15.10 ± 1.82^b2^	36.35 ± 0.04	34.13 ± 0.08^b3^	−6.10 ± 0.22^b3^	25.00 ± 0.93	22.67 ± 0.76	−9.14 ± 2.07^b3^
200 mg/kg AF	54.17 ± 0.83	46.67 ± 1.31^b3^	−13.75 ± 2.67^b2^	36.45 ± 0.11	34.48 ± 0.07^b3^	−5.39 ± 0.21^b3^	25.50 ± 1.38	23.50 ± 1.23	−7.76 ± 0.82^b2^
400 mg/kg AF	52.00 ± 0.97	45.17 ± 1.30^b3^	−13.01 ± 2.80^b1^	36.33 ± 0.06	34.73 ± 0.08^b3,c1^	−4.40 ± 0.14^a2,b3^	25.17 ± 1.45	23.67 ± 1.05	−5.57 ± 1.45^a1^
10 ml/kg 2% *T* 80^*∗*^	53.17 ± 2.24	44.17 ± 1.22	−16.32 ± 3.57	36.53 ± 0.11	34.08 ± 0.18	−6.71 ± 0.22	26.83 ± 1.01	24.00 ± 0.68	−10.37 ± 1.38
CHQ 25 mg/kg^*∗*^	51.83 ± 2.57	50.67 ± 2.35^a1^	−1.60 ± 4.62^a2^	36.53 ± 0.09	36.50 ± 0.09^a3^	−0.09 ± 0.06^a3^	24.83 ± 1.05	25.00 ± 1.15	0.59 ± 0.60^a3^
100 mg/kg DF	56.17 ± 2.24	48.33 ± 1.28	−13.53 ± 2.73^a1^	36.50 ± 0.09	34.60 ± 0.09^a1,b3,e3^	−5.21 ± 0.01^a3,b3,e3^	24.67 ± 1.23	23.33 ± 1.12	−5.34 ± 0.70^a3,b2^
200 mg/kg DF	53.83 ± 1.14	49.33 ± 1.28	−8.12 ± 3.34^a1^	36.58 ± 0.08	35.17 ± 0.09^a3,b3,c1^	−3.87 ± 0.09^a3,b3,c3^	24.33 ± 1.33	23.50 ± 1.26	−3.37 ± 0.70^a3,b2^
400 mg/kg DF	52.17 ± 1.30	48.17 ± 1.19^a1^	−5.10 ± 2.56^a2^	36.53 ± 0.12	35.50 ± 0.13^a3,b3,c3^	−2.83 ± 0.07^a3,b3,d3^	24.67 ± 1.26	24.00 ± 1.06	−2.52 ± 0.80^a3^
100 mg/kg HF	53.50 ± 1.82	44.50 ± 1.77	−16.89 ± 0.62^b1^	36.53 ± 0.09	34.23 ± 0.09^b3^	−6.30 ± −6.34^b3,d2^	25.50 ± 1.18	22.83 ± 1.05	−10.42 ± 1.09^b3^
200 mg/kg HF	54.00 ± 2.39	46.00 ± 2.03	−14.18 ± 4.70	36.50 ± 0.15	34.43 ± 0.16^b3^	−5.66 ± −5.91^a1,b3,e2^	24.17 ± 1.58	22.00 ± 0.93	−8.24 ± 2.43^b2^
400 mg/kg HF	56.67 ± 1.45	49.33 ± 1.36	−12.86 ± 1.89	36.47 ± 0.09	34.67 ± 0.09^a1,b3^	−4.94 ± −4.97^a2,b3,c3^	25.50 ± 1.18	23.67 ± 0.76	−6.89 ± 1.45^b1^

Data are expressed as mean ± SEM; *n* = 6, *a* = compared to the negative control, *b* = compared to the positive control, *c* = compared to 100 mg/kg, *d* = compared to 200 mg/kg, *e* = compared to 400 mg/kg, ^1^*p* < 0.05, ^2^*p* < 0.01, ^3^*p* < 0.001, ^*∗*^ = negative and positive controls for dichloromethane and hexane fractions, SEM = standard error of the mean, *D*0 = day 0, *D*4 = day 4, DW = distilled water, CE = crude extract, AF = aqueous fraction, DF = dichloromethane fraction, HF = hexane fraction, *T* 80 = tween 80, and CHQ = chloroquine.

**Table 4:** Effects of crude extract and dichloromethane fraction on the parasitemia level and mean survival time in the curative test.

Groups	% Parasitemia					% Inhibition	Mean survival time
	D3	D4	D5	D6	D7		
10 ml/kg DW	20.50 ± 0.76	22.67 ± 0.67	24.50 ± 0.56	26.17 ± 0.70	28.33 ± 0.67	0.00	8.00 ± 0.58
CHQ 25 mg/kg	21.67 ± 0.76	19.50 ± 0.67^a1,c3^	13.33 ± 0.61^a3^	5.17 ± 0.60^a3^	0.00 ± 0.00^a3^	100.00	30.00 ± 0.00^a3^
100 mg/kg CE	22.67 ± 1.02	22.33 ± 0.80^d1,e2^	22.00 ± 0.73^a1,b3^	21.67 ± 0.84^a2,b3,e2^	18.50 ± 0.89^a3,b3,e3^	34.70	13.17 ± 0.60^a3,b3,e3^
200 mg/kg CE	23.00 ± 1.13	22.17 ± 1.05	21.50 ± 0.89^a1,b3^	20.17 ± 0.79^a3,b3,e1^	16.17 ± 0.79^a3,b3,e3^	42.93	15.17 ± 0.60^a3,b3,e1^
400 mg/kg CE	22.50 ± 0.67	21.67 ± 0.56	19.33 ± 0.61^a3,b3^	17.17 ± 0.54^a3,b3^	10.17 ± 0.54^a3,b3^	64.10	17.67 ± 0.42^a3,b3^
10 ml/kg 2% *T* 80^*∗*^	20.00 ± 0.58	22.17 ± 0.79	23.83 ± 0.60	25.67 ± 0.84	27.17 ± 0.60	0.00	7.67 ± 0.33
CHQ 25 mg/kg^*∗*^	21.33 ± 0.76	19.00 ± 0.68^a1^	12.67 ± 0.76^a3^	4.83 ± 0.48^a3^	0.00 ± 0.00^a3^	100.00	30.00 ± 0.00^a3^
100 mg/kg DF	22.50 ± 1.12	21.67 ± 0.92^d1,e2^	21.50 ± 0.43^a2,b3,e2^	20.67 ± 0.61^a3,b3,e3^	18.33 ± 0.67^a3,b3,d3^	32.54	13.33 ± 0.49^a3,b3,d3^
200 mg/kg DF	22.00 ± 1.12	21.00 ± 0.77	20.17 ± 0.79^a2,b3^	18.67 ± 0.80^a3,b3,e1^	14.67 ± 0.71^a3,b3,e3^	46.00	18.17 ± 0.79^a3,b3,e3^
400 mg/kg DF	21.00 ± 0.68	19.50 ± 0.56	17.50 ± 0.76^a3,b3^	15.17 ± 0.79^a3,b3^	8.17 ± 0.48^a3,b3,c3^	69.93	21.33 ± 0.42^a3,b3,c3^

Data are expressed as mean ± SEM; *n* = 6, *a* = compared to the negative control, *b* = compared to the positive control, *c* = compared to 100 mg/kg dose, *d* = compared to 200 mg/kg dose, *e* = compared to 400 mg/kg dose, ^1^*p* < 0.05, ^2^*p* < 0.01, ^3^*p* < 0.001, ^*∗*^ = negative and positive controls for dichloromethane fraction, *D*0 = day 0, *D*4 = day 4, DW = distilled water, CE = crude extract, DF = dichloromethane fraction, *T* 80 = tween 80, and CHQ = chloroquine.

**Table 5:** Packed cell volume (PCV), weight, and temperature for the crude extract and dichloromethane fraction of the stem bark of *Acacia tortilis* in the curative test.

Groups	PCV			Rectal temperature (°C)			Body weight (g)		
	D3	D7	% Change	D3	D7	% Change	D3	D7	% Change
10 ml/kg DW	50.00 ± 1.29	40.33 ± 1.47	−9.67 ± 1.56	35.27 ± 0.27	33.58 ± 0.23	−1.68 ± 0.25	19.00 ± 1.37	16.00 ± 1.06	−3.00 ± 0.37
CHQ 25 mg/kg	50.50 ± 0.76	49.67 ± 0.66^a3^	−0.83 ± 1.66^a3^	35.92 ± 0.23	36.60 ± 0.15^a3^	0.68 ± 0.26^a3^	24.17 ± 0.98	24.00 ± 0.85^a3^	−0.59 ± 0.59^a2^
100 mg/kg CE	51.33 ± 0.66	43.83 ± 1.51^b2^	−7.50 ± 1.02^b2^	35.23 ± 0.25	33.45 ± 0.12^b3,d2^	−1.78 ± 0.28^b3^	24.67 ± 1.02	22.00 ± 0.89^a2^	−2.67 ± 0.42
200 mg/kg CE	50.67 ± 0.49	46.50 ± 0.76^b1^	−4.17 ± 1.07^a2^	35.78 ± 0.17	34.47 ± 0.35^b3^	−1.32 ± 0.19^a1,b3^	24.00 ± 1.43	23.33 ± 1.35^a3^	−2.71 ± 0.88
400 mg/kg CE	48.33 ± 0.80	44.83 ± 0.79^b1^	−3.50 ± 0.99^a2^	35.78 ± 0.09	34.75 ± 0.15^b3,c2^	−1.03 ± 0.11^a1,b3^	24.83 ± 0.87	22.83 ± 0.70^a3^	−2.00 ± 0.68^a1^
10 ml/kg 2% *T* 80^*∗*^	47.17 ± 2.24	39.17 ± 2.54	−17.16 ± 2.71	35.70 ± 0.25	34.10 ± 0.26	−4.48 ± 0.03	21.67 ± 0.95	19.83 ± 0.98	−8.57 ± 0.90
CHQ 25 mg/kg^*∗*^	46.83 ± 2.57	47.83 ± 2.84^a1^	2.17 ± 0.69^a3^	36.23 ± 0.09	37.23 ± 0.08^a3^	2.76 ± 0.00^a3^	26.83 ± 1.04	26.67 ± 1.05^a3^	−0.62 ± 0.61^a3^
100 mg/kg DF	47.17 ± 1.30	46.17 ± 1.40	−2.13 ± 0.55^a3^	35.75 ± 0.09	34.35 ± 0.09^b3^	−3.92 ± 0.01^a3,b3,d3^	22.33 ± 1.02	20.33 ± 1.02^b3^	−9.05 ± 0.42^b3,e1^
200 mg/kg DF	49.83 ± 1.14	48.83 ± 1.30	−2.01 ± 0.56^a3^	35.38 ± 0.08	34.08 ± 0.07^b3^	−3.67 ± 0.01^a3,b3,e3^	22.33 ± 0.95	21.00 ± 1.06^b2^	−6.11 ± 1.10^b3^
400 mg/kg DF	52.17 ± 2.24	50.17 ± 2.12	−1.93 ± 0.45^a3,b1^	35.23 ± 0.12	34.13 ± 0.12^b3^	−3.12 ± 0.01^a3,b3,c3^	24.33 ± 0.84	23.00 ± 0.68	−5.39 ± 0.69^a1,b2^

Data are expressed as mean ± SEM; *n* = 6, *a* = compared to the negative control, *b* = compared to the positive control, *c* = compared to 100 mg/kg dose, *d* = compared to 200 mg/kg dose, *e* = compared to 400 mg/kg dose, ^1^*p* < 0.05, ^2^*p* < 0.01, ^3^*p* < 0.001, ^*∗*^ = negative and positive controls for the dichloromethane fraction, *D*0 = day 0, *D*4 = day 4, DW = distilled water, CE = crude extract, DF = dichloromethane fraction, *T* 80 = tween 80, and CHQ = chloroquine.

**Table 6:** Effects of the crude extract and solvent fractions of *Acacia tortilis* on the parasitemia level and mean survival time in the prophylactic test.

Treatment and doses	% Parasitemia	% Suppression	Mean survival time (days)
10 ml/kg DW	29.00 ± 1.06	—	7.33 ± 1.50
CHQ 25 mg/kg	0.33 ± 0.33^a3^	98.86	29.50 ± 1.22^a3^
100 mg/kg CE	20.50 ± 1.40^a3,b3^	29.31	11.33 ± 1.63^a2,b3,e3^
200 mg/kg CE	17.83 ± 1.13^a3,b3^	38.51	12.83 ± 0.98^a3,b3,e1^
400 mg/kg CE	15.33 ± 0.55^a3,b3,c2^	47.13	15.83 ± 1.72^a3,b3^
10 ml/kg 2% *T* 80^*∗*^	31.00 ± 0.57	—	6.67 ± 0.49
CHQ 25 mg/kg^*∗*^	0.00 ± 0.00^a3^	100	30.00 ± 0.00^a3^
100 mg/kg DF	24.17 ± 1.07^a3,b3^	22.03	9.50 ± 0.67^a2,b3^
200 mg/kg DF	19.00 ± 1.34^a3,b3^	38.70	16.33 ± 0.84^a3,b3^
400 mg/kg DF	15.83 ± 0.87^a3,b3^	48.93	17.50 ± 1.47^a3,b2^

Data are expressed as mean ± SEM; *n* = 6, *a* = compared to the negative control, *b* = compared to the positive control, *c* = compared to 100 mg/kg dose, *d* = compared to 200 mg/kg dose, *e* = compared to 400 mg/kg dose, ^1^*p* < 0.05, ^2^*p* < 0.01, ^3^*p* < 0.001, ^*∗*^ = negative and positive controls for the dichloromethane fraction, *D*0 = day 0, *D*4 = day 4, DW = distilled water, CE = crude extract, DF = dichloromethane fraction, *T* 80 = tween 80, and CHQ = chloroquine.

**Table 7:** Effects of *Acacia tortilis* on packed cell volume (PCV), weight, and temperature for the crude extract and dichloromethane fraction of the stem bark of *Acacia tortilis* in the prophylactic test.

Groups	PCV			Rectal temperature (°C)			Body weight (g)		
	D0	D7	% Change	D0	D7	% Change	D0	D7	% Change
10 ml/kg DW	50 .00 ± 1.92	43.50 ± 1.81	−13.00 ± 1.21	36.11 ± 0.12	34.52 ± 0.21	−4.40 ± 0.14	25.34 ± 1.64	22.54 ± 1.32	−11.05 ± 0.83
CHQ 25 mg/kg	48.40 ± 1.03	49.50 ± 1.31^a1^	2.27 ± 0.98^a3^	36.55 ± 0.17	36.81 ± 0.14	0.71 ± 0.08^a2^	23.86 ± 1.42	23.98 ± 0.12	0.50 ± 0.24^a3^
100 mg/kg CE	53.80 ± 1.08	48.30 ± 1.02	−10.22 ± 0.75^b2^	37.20 ± 0.16	36.13 ± 0.13	−2.88 ± 0.11^b1^	24.42 ± 0.54	22.28 ± 0.83	−8.75 ± 0.15^b2^
200 mg/kg CE	52.90 ± 0.91	48.20 ± 0.74	−8.88 ± 0.25^b2,a1^	36.65 ± 0.24	35.85 ± 0.17	−2.18 ± 0.06	27.21 ± 0.68	25.19 ± 0.65	−7.42 ± 0.18^b1^
400 mg/kg CE	53.00 ± 1.66	49.50 ± 1.56^a1^	−6.60 ± 1.33^b1,a2^	36.45 ± 0.31	35.82 ± 0.26	−1.73 ± 0.16^a1^	25.68 ± 1.08	24.33 ± 1.13	−5.25 ± 0.32^a1^
10 ml/kg 2% *T* 80^*∗*^	48.50 ± 1.13	42.40 ± 1.15	−12.58 ± 1.10	36.44 ± 0.34	34.85 ± 0.25	−4.36 ± 0.18	26.83 ± 0.94	23.91 ± 0.76	−10.85 ± 0.41
CHQ 25 mg/kg^*∗*^	48.20 ± 1.00	49.00 ± 1.05^a1^	1.66 ± 0.56^a3^	36.24 ± 0.14	36.43 ± 0.12	0.52 ± 0.07^a2^	23.90 ± 0.87	24.03 ± 1.03	0.55 ± 0.58^a3^
100 mg/kg DF	53.20 ± 1.24	48.32 ± 1.14	−9.17 ± 1.02^b3^	36.75 ± 0.22	35.83 ± 0.19	−2.50 ± 0.12^b1^	24.82 ± 1.48	22.78 ± 1.26	−8.20 ± 0.43^b2^
200 mg/kg DF	51.60 ± 1.29	47.73 ± 1.17	−7.50 ± 0.88^a1,b2^	36.90 ± 0.27	36.19 ± 0.21	−1.92 ± 0.16	25.55 ± 1.35	23.81 ± 1.07	−6.82 ± 0.96^b1^
400 mg/kg DF	48.80 ± 1.61	46.26 ± 1.57	−5.20 ± 1.08^a2,b1^	36.60 ± 0.31	36.01 ± 0.29	−1.61 ± 0.20^a1^	26.25 ± 1.32	24.93 ± 1.28	−5.04 ± 0.92^a2^

Data are expressed as mean ± SEM; *n* = 6, *a* = compared to the negative control, *b* = compared to the positive control, *c* = compared to 100 mg/kg dose, *d* = compared to 200 mg/kg dose, *e* = compared to 400 mg/kg dose, ^1^*p* < 0.05, ^2^*p* < 0.01, ^3^*p* < 0.001, ^*∗*^ = negative and positive controls for the dichloromethane fraction, *D*0 = day 0, *D*4 = day 4, DW = distilled water, CE = crude extract, DF = dichloromethane fraction, *T* 80 = tween 80, and CHQ = chloroquine.

## Data Availability

The datasets are available from the corresponding author upon reasonable request.

## Abbreviations

PCV: Packed cell volume
OECD: Organization for economic cooperation and development
RBC: Red blood cell
MST: Mean survival time
SEM: Standard error of the mean.
